# Analysis of Cardiac Adverse Reactions Caused by Different Doses of Adriamycin Chemotherapy in Patients with Breast Cancer

**DOI:** 10.1155/2022/1642244

**Published:** 2022-02-15

**Authors:** Guangwen Hu, Daxin Wang

**Affiliations:** ^1^Department of Cardiology, Haining Central Hospital, Haining, Zhejiang 314400, China; ^2^Department of Cardiovascular Medicine, Yangzhou University, Yangzhou, Jiangsu 225000, China

## Abstract

**Purpose:**

This paper is aimed at studying the adverse reactions of breast cancer patients after chemotherapy with different doses of adriamycin.

**Methods:**

122 breast cancer patients undergoing mastectomy in the Haining Central Hospital from June 2018 to June 2020 were selected as the research objects. Patients were divided into control group and study group according to the different dose of adriamycin given to patients during chemotherapy. Patients in the control group received intravenous drip of adriamycin at 50 mg/m^2^. Patients in the study group were given intravenous drip at 75 mg/m^2^. Patients in both the groups started intravenous drip of cyclophosphamide 500 mg/m^2^ on the first day of chemotherapy, and chemotherapy for 21 days was a cycle. A total of 6 cycles were carried out. Abnormal electrocardiograph (ECG) is compared between the two groups. Myocardial enzyme and oxidative stress indicators were tested, and Doppler ultrasound examination was conducted.

**Results:**

After chemotherapy, the abnormal rate of ECG in the study group was 56.46%, which was significantly higher than that in the control group (46.67%). After chemotherapy, the indexes of myocardial enzymes and oxidative stress increased, while superoxide dismutase (SOD) decreased significantly, and the differences were statistically significant. At the end of chemotherapy, the differences of serum myocardial enzymes and oxidative stress indexes in the study group were higher than those in the control group. After chemotherapy, there was no significant difference between left ventricular ejection fraction (LVEF) and Sa in the study group and the control group, but Ea in the study group was higher than that in the control group and E/Ea was lower than that in the control group.

**Conclusion:**

High-dose adriamycin chemotherapy is more likely to cause accumulation of cardiotoxicity, resulting in decreased cardiac function and cardiac injury in breast cancer patients.

## 1. Introduction

The incidence and mortality of breast cancer in female patients are relatively high, which seriously threatens the life safety of patients [1]. However, with the continuous improvement of current medical technology, the survival rate of patients can be improved to a large extent. As a basic chemotherapy drug for adenocarcinoma, adriamycin milk has a definite effect on breast cancer [2]. Although adriamycin has a good effect on chemotherapeutic drugs for breast cancer patients, studies have shown that adriamycin chemotherapy can cause adverse cardiac reactions in breast cancer patients, which may cause some effects on the cardiac function of patients, and even cause heart failure [3]. Cardiotoxicity of adriamycin in different patients may be related to age, disease, dose, and cumulative dose of patients [4]. In this study, 122 cases of breast cancer patients treated with different doses of adriamycin chemotherapy in our hospital were studied, and the effects of adriamycin chemotherapy on cardiac adverse reactions in breast cancer patients were statistically analyzed.

## 2. Materials and Methods

### 2.1. General Data

A total of 122 breast cancer patients who received mastectomy and were about to receive adriamycin chemotherapy in our hospital from June 2018 to June 2020 were selected as the research subjects. According to the different doses of adriamycin given to patients during chemotherapy, the patients were divided into a low-dose group (60 cases) and a high-dose group (62 cases). There was no statistical significance in the basic data between the two groups (*p* > 0.05), as shown in Table 1.

Inclusion criteria: (1) breast cancer diagnosed by pathology after surgery; (2) patients who had not received any treatment for breast cancer except surgery before inclusion treated with AC combined with chemotherapy (doxorubicin + cyclophosphaamide needle); women over 18 years of age with breast cancer after mastectomy and chemotherapy; (3) no significant abnormality in blood routine, liver, and kidney function, and no abnormality in ECG and cardiac function evaluation before chemotherapy.

Exclusion criteria: (1) patients who had previously received antitumor therapy other than surgery; (2) lactation and pregnant patients; (3) congenital heart disease or coronary heart disease, hypertension, and other past histories. All patients in this study gave informed consent and were reviewed by the Medical Ethics Committee with the Approval No. 2018–21.

## 3. Methods

Two groups of patients were treated with adriamycin-based combined chemotherapy regimen: adriamycin (manufacturer: Pfizer, approval number: H20130186) + cyclophosphamide injection (manufacturer: Shanxi Pude Pharmaceutical Co., Ltd., approval number: H14023686) for chemotherapy. The two groups of patients started chemotherapy on the 6th day after surgery, and the control group received intravenous infusion of adriamycin at 50 mg/m^2^. Patients in the study group received 75 mg/m^2^ intravenous infusion. Both groups received cyclophosphamide 500 mg/m^2^ intravenous infusion on day 1, 21 days as a cycle. There were 6 cycles of chemotherapy.

### 3.1. Observation Index

ECG abnormalities were occurred. The ECG monitored by the ECG instrument (Japan Optoelectronics, ECG-1250C) before and after chemotherapy was compared between the two groups. Atrial premature beats, ventricular premature beats, supraventricular tachycardia, sinus tachycardia, bradycardia, ST-T changes, QT-QTC extension, QRS low voltage, bundle branch block, and so on were statistically analyzed. Cardiac enzyme test results and oxidative stress indexes before and after chemotherapy in the two groups were compared, mainly including aspartate aminotransferase (AST), lactate dehydrogenase (LDH), creatine phosphokinase isoenzyme (CPK-MB), *a*-hydroxybutyrate dehydrogenase (*α*-HBDH), and creatine phosphokinase (CPK). Serum superoxide dismutase (SOD) and thiobarbituric acid were used to determine serum malondialdehyde (MDA). Doppler ultrasonography (Philips IE33) before and after chemotherapy was compared between the two groups. The LVEF is calculated; peak systolic velocity (Sa), early diastolic blood flow velocity (*E*), and early diastolic motion velocity (Ea) of the left atrioventricular annulus at 2 loci were measured and calculated, and E/Ea at 2 loci were calculated.

### 3.2. Statistical Processing

SPSS 22.0 statistical software was used for data processing. Measurement data were expressed as *x* ± *s*, and the *t* -test was performed. Counting data were expressed as example (%), and the X^2^ test was performed.

## 4. Results

### 4.1. Complete Enrollment of Patients and General Conditions after Chemotherapy

Of the 129 patients, 2 were excluded from the group with severe myelosuppression, and 5 were lost to followup for other reasons. The remaining 122 cases were analyzed statistically. The remaining 115 patients all completed the scheduled 6 cycles of chemotherapy; there were 82 cases of gastrointestinal reaction (67.21%), 43 cases of mild myelosuppression (35.25%), and 26 cases of palpitation (21.31%).

### 4.2. Comparison of Abnormal Electrocardiogram in the Two Groups before Chemotherapy

The results showed no abnormal conditions in both the groups. After 6 cycles of chemotherapy, the abnormal rate of electrocardiogram in the study group was 56.46%, which was significantly higher than that in the control group (46.67%), and the difference was statistically significant (*P* < 0.05), as shown in Table 2.

### 4.3. Changes of Serum Myocardial Enzymes and Oxidative Stress Indexes in the Two Groups before and after Chemotherapy

Comparison of the levels of myocardial enzyme indexes AST, LDH, CK, CK-MB, and *a*-HBDH in the two groups after chemotherapy was increased, the oxidative stress index MDA was increased, and SOD was significantly decreased, and the differences were statistically significant. The difference of serum myocardial enzymes and oxidative stress indexes in the study group was higher than that in the control group, and the difference was statistically significant (*P* < 0.05), as shown in Table 3.

### 4.4. Comparison of Doppler Ultrasound Indications between the Two Groups

There were no significant differences in LVEF, Ea, Sa, and E/Ea before chemotherapy between the two groups. After chemotherapy, there was no statistically significant difference in LVEF and Sa between the study group and the control group. Ea in the study group was higher than that in the control group, while E/Ea was lower than that in the control group. The difference was statistically significant (*P* < 0.05), as shown in Table 4.

## 5. Discussion

Currently, the main treatment for breast cancer is surgical treatment, and adjuvant chemotherapy is an important guarantee to ensure the survival rate of patients [5, 6]. Adriamycin has been proved to be effective in chemotherapy for breast cancer patients and has gradually become the drug of choice in chemotherapy for breast cancer patients. It can not only destroy the protein and cell wall of tumor cells but also has an inhibitory effect on their DNA ligase, thus effectively inhibiting the growth of tumor cells [7–9]. However, its myelosuppression and cardiotoxicity should not be ignored, especially cardiotoxicity, which may lead to delayed progression, thus restricting the application of doxorubicins [10, 11]. In this study, the adverse cardiac reactions caused by different doses of adriamycin chemotherapy in breast cancer patients were deeply analyzed to understand the cardiotoxicity characteristics of different concentrations of adriamycin so as to provide a basis for the adjustment of treatment regimens for patients with adriamycin and improve the treatment effect of patients.

The results of this study showed that the abnormal rate of ECG in the study group after chemotherapy was 56.46% significantly higher than that in the control group (46.67%). Myocardial enzymology is an important indicator for the diagnosis of myocardial injury, but it lacks tissue specificity and exists in all tissues and organs of the human body. At present, serum CK-MB and other indicators are recommended to be detected clinically [12]. Studies have shown that the cardiotoxicity of anthracycline chemotherapies is mainly due to the chelation of adriamycin with iron ions, which stimulates the release of Ca^2+^, affects the protein gene expression, destroys the balance of Ca^2+^, produces excessive oxygen free radicals, damages myocardial cells, and causes delayed cardiac injury. SOD and MDA are commonly used indexes to evaluate the oxidative stress level [13]. This study showed that after chemotherapy, the myocardial enzyme index and the oxidative stress index of MDA increased and SOD decreased significantly in both the groups, and the differences were statistically significant. At the end of chemotherapy, serum myocardial enzyme and oxidative stress indexes in the research group were higher than those in the control group, and the differences were statistically significant. It is also further confirmed that a high dose of adriamycin can reduce the ability of free radical scavenging in patients so that the body of chemotherapy patients produce excessive lipid peroxidation products and then cause damage to cardiomyocytes. When the myocardium is seriously damaged, LVEF will have abnormal changes, which is one of the commonly used clinical indicators to detect the overall damaged function of the heart, but it is not suitable for the early detection of myocardial damage. The systolic function parameter SA and diastolic function parameter EA, E/EA can be detected by Doppler ultrasound to detect the systolic and diastolic function of the patient's left ventricle. The study showed that there was no statistically significant difference in LVEF and SA in the study group after chemotherapy compared with the control group, while Ea was higher than the control group and E/Ea was lower than the control group, and the difference was statistically significant.

High dose adriamycin chemotherapy is more likely to cause accumulation of cardiotoxicity, resulting in decreased cardiac function and cardiac injury in breast cancer patients. Therefore, we need to take appropriate dose to ensure the efficacy of chemotherapy and reduce the cardiotoxicity caused by doxorubicin as much as possible.

## Figures and Tables

**Table 1:** Comparison of general data between two groups of patients.

Groups	Numbers	Age	Body mass index	*Cancer* classification		Stage			
				Noninvasive carcinoma	Invasive carcinoma	IIA	IIB	IIIA	IIIB
Control group	60	55.62 ± 5.37	22.58 ± 1.35	28	32	15	21	13	11
Experiment group	62	53.59 ± 6.67	23.04 ± 1.13	29	31	15	22	14	11
*p*		>0.05	>0.05	>0.05		>0.05			

**Table 2:** Comparison of abnormal ECG after chemotherapy between two groups.

Groups	n	Atrial premature beats	Ventricular premature beat	Supraventricular tachycardia	Nodal tachycardia	Sinus bradycardia	ST-T change	QT-QTc prolong	QRS low voltage	Interventricular heart-block	Abnormal rate
Control group	60	6 (10)	4 (6.67)	0 (0.00)	4 (6.67)	4 (6.67)	2 (3.23)	3 (5.00)	3 (5.00)	2 (3.23)	28 (46.67)
Experiment group	62	7 (11.3)	5 (8.06)	2 (3.22)	7 (11.3)	4 (6.45)	3 (4.84)	3 (4.84)	2 (3.22)	2 (3.22)	35 (56.45)
X^2^											6.678
*p*											0.01

**Table 3:** Comparison of changes of serum myocardial enzymes and oxidative stress indexes between two groups before and after chemotherapy (*X* ± *S*).

Index	Control group			Experiment group			t	*p*
	Before chemotherapy	After chemotherapy	Δ^*∗*^	Before chemotherapy	After chemotherapy	Δ^*∗*^		
AST (U/L)	99.82 ± 27.42	115.63 ± 36.38	16.32 ± 3.26^*∗*^	98.36 ± 24.62	135.26 ± 38.63	36.52 ± 5.32^*∗*^	9.52	<0.05
LDH (U/L)	151.37 ± 33.64	163.52 ± 38.52	11.35 ± 2.89^*∗*^	152.01 ± 32.85	169.85 ± 35.65	18.62 ± 2.36^*∗*^	7.98	<0.05
CK (U/L)	107.67 ± 29.73	108.63 ± 29.58	1.35 ± 0.28^*∗*^	107.52 ± 29.33	118.63 ± 31.23	15.28 ± 2.08^*∗*^	10.68	<0.05
CK-MB (U/L)	18.66 ± 6.54	20.03 ± 6.66	2.33 ± 0.59^*∗*^	18.72 ± 6.48	28.65 ± 7.62	12.32 ± 2.65^*∗*^	10.66	<0.05
*α*-HBDH (U/L)	109.66 ± 38.26	125.36 ± 42.55	17.63 ± 2.21^*∗*^	109.75 ± 38.42	132.56 ± 45.36	23.62 ± 4.25^*∗*^	9.98	<0.05
SOD (U/mL)	169.21 ± 9.56	136.65 ± 8.25	-30.25 ± 5.38^*∗*^	169.21 ± 9.56	115.36 ± 12.25	-48.63 ± 8.63^*∗*^	12.35	<0.05
MDA (nmol/L)	3.95 ± 0.56	12.36 ± 0.85	7.56 ± 1.86^*∗*^	3.95 ± 0.56	18.63 ± 3.25	15.52 ± 2.63^*∗*^	6.32	<0.05

Note: Δ represents the change of indicators after chemotherapy compared with before chemotherapy, that is after chemotherapy–before chemotherapy; ^*∗*^ represents the comparison between the study group and the control group after chemotherapy.

**Table 4:** Comparison of Doppler ultrasound examination indexes between the two groups (*X* ± *S*).

	Control group			Experiment group			t	*p*
	Before chemotherapy	After chemotherapy	Δ^*∗*^	Before chemotherapy	After chemotherapy	Δ^*∗*^		
LVEF (%)	0.62 ± 0.07	0.60 ± 0.05	0.02 ± 0.01^*∗*^	0.61 ± 0.08	0.63 ± 0.06	0.02 ± 0.01^*∗*^	0.635	>0.05
Sa (cm/s)	8.92 ± 0.85	8.89 ± 0.88	0.03 ± 0.01^*∗*^	8.93 ± 0.88	8.92 ± 0.85	0.02 ± 0.01^*∗*^	0.752	>0.05
Ea (cm/s)	11.32 ± 2.23	13.63 ± 1.89	2.03 ± 0.32^*∗*^	11.36 ± 2.20	15.96 ± 2.01	4.53 ± 0.36^*∗*^	6.325	<0.05
E/Ea	5.66 ± 0.83	5.38 ± 0.75	-0.25 ± 0.05^*∗*^	5.62 ± 0.85	5.26 ± 0.66	-0.41 ± 0.08^*∗*^	3.256	<0.05

Note: Δ represents the change of indicators after chemotherapy compared with before chemotherapy, that is after chemotherapy–before chemotherapy; ^*∗*^ represents the comparison between the study group and the control group after chemotherapy.

## Data Availability

Data used to support the findings of this study are available on reasonable request from the corresponding author.
